This article has been retracted.

# *ALDH2* and *ADH1* Genetic Polymorphisms May Contribute to the Risk of Gastric Cancer: A Meta-Analysis

**DOI:** 10.1371/journal.pone.0088779

**Published:** 2014-03-14

**Authors:** He-Ling Wang, Ping-Yi Zhou, Peng Liu, Yu Zhang

**Affiliations:** Department of General Surgery, Shengjing Hospital of China Medical University, Shenyang, P. R. China; The University of Hong Kong, China

## Abstract

**Aim:**

We conducted a meta-analysis of case-control studies to determine whether *ALDH2*, *ADH1* and *ADH2* genetic polymorphisms contribute to the pathogenesis of gastric cancer.

**Methods:**

The PubMed, CISCOM, CINAHL, Web of Science, Google Scholar, EBSCO, Cochrane Library, and CBM databases were searched for relevant articles published before November 1st, 2013 without any language restrictions. Meta-analysis was conducted using the STATA 12.0 software. We calculated crude odds ratios (ORs) with their 95% confidence intervals (95%CI) to evaluate their relationships under five genetic models. Seven case-control studies with a total of 2,563 gastric cancer patients and 4,192 healthy controls met the inclusion criteria. Nine common polymorphisms were evaluated, including rs671, rs16941667 and rs886205 in the *ALDH2* gene, rs1230025, rs13123099, rs698 and rs1693482 in the *ADH1* gene, and rs1229984 and rs17033 in the *ADH2* gene.

**Results:**

The results of our meta-analysis suggested that *ALDH2* genetic polymorphisms might be strongly correlated with an increased risk of gastric cancer (allele model: OR  = 1.21, 95%CI: 1.11∼1.32, *P*<0.001; dominant model: OR  = 1.23, 95%CI: 1.09∼1.39, *P* = 0.001; respectively), especially for rs671 polymorphism. Furthermore, we observed significant associations between *ADH1* genetic polymorphisms and an increased risk of gastric cancer (allele model: OR  = 1.21, 95%CI: 1.08∼1.36, *P* = 0.001; dominant model: OR  = 10.52, 95%CI: 3.04∼36.41, *P*<0.001; respectively), especially for rs1230025 polymorphism. Nevertheless, no positive relationships were found between *ADH2* genetic polymorphisms and gastric cancer risk (all *P*>0.05).

**Conclusion:**

The current meta-analysis suggests that *ALDH2* and *ADH1* genetic polymorphisms may play crucial roles in the pathogenesis of gastric cancer. However, *ADH2* genetic polymorphisms may not be important dominants of susceptibility to gastric cancer.

## Introduction

Gastric cancer is one of the most frequently diagnosed digestive tract cancers, which is often asymptomatic or with nonspecific signs and symptoms in its early stage resulting in relatively poor prognosis [1]. The incidence of gastric cancer varies remarkably around the world with predominant prevalence in some Asian, Eastern European countries and lower rates in Africa, Oceania, North America, and Brazil [2]. Even though the past decades have witnessed a major decrease in incidence and mortality of gastric cancer throughout the world, gastric cancer remains the fourth common cancer worldwide and the second leading cause of cancer mortality responsible for about 800,000 deaths worldwide per year [3]. Previous studies have shown that helicobacter pylori infection may be the strongest established risk factor for 65∼80% of gastric cancer which makes gastric cancer the only bacterium-associated human malignancy [4], [5]. Furthermore, environmental factors, dietary habits and genetic susceptibility have also been demonstrated to play important roles in the etiology of gastric cancer [6]. It has been widely accepted that ethanol consumption appears to be a strong risk factor for the occurrence and development of certain types of cancers [7], [8]. It is well established that ethanol is oxidized first to acetaldehyde and then to acetate by alcohol dehydrogenases (ADHs) and aldehyde dehydrogenases (ALDHs) in the liver and upper gastrointestinal [9]. Acetaldehyde is recognized to be carcinogenic in animals and suspected to has the same function on human beings, whose accumulation in the blood may cause adverse symptoms of facial flushing, palpitation and headache [10]. Epidemiologic evidence has shown that alcohol drinking could cause DNA damage in stomach [11], [12]. Especially when the human body is flooded with exogenous ethanol, the concentrations of acetaldehyde produced vastly exceed the trace amounts and theoretically conferring a correspondingly high risk of tumorigenesis [13].

The ADH isoenzymes generally refer to a metabolic barrier against orally self-administer ethanol and also against ethanol produced from carbohydrates through fermentation of bacterial [14], [15]. ADH1 and ADH2, two well-known members of ADH family, mainly expressed in the liver but also the gastric mucosa, is significantly responsible for the partially metabolism of orally ingested alcohol, namely, in the conversion of ethanol to its carcinogenic metabolite, acetaldehyde, particularly during the elimination phase [16]–[18]. Both *ADH1* and *ADH2* genes are located in a cluster on chromosome 4q22∼23 [19]. ALDH2, belonging to a low-Km mitochondrial ALDH and expressing in the liver as well as stomach, is the second enzyme to eliminate most of the acetaldehyde generated during alcohol metabolism *in vivo* [20]. Human *ALDH2* gene is located on chromosome 12q24.2 and composed of 13 exons, spanning 46,031 bp [21]. ALDH2 is usually thought to dispose of acetaldehyde to non-toxic acetate generated during the metabolism of ethanol, in contrast, while reduced expression of ALDH2 will induce a marked increase in blood acetaldehyde in individuals who consume ethanol [22], [23].

Genetic variants in *ALDH2/ADH1/ADH2* genes may contribute to alteration in alcohol metabolism which may resulting in the promotion of ethanol oxidation, and may be closely associated with the inhibition of acetaldehyde oxidation, conducing to the accumulation of acetaldehyde [14], [24], [25]. Therefore, it is hypothesized that genetic polymorphisms in the *ALDH2/ADH1/ADH2* genes may be strongly correlated with the susceptibility to gastric cancer [16], [26], [27]. Nevertheless, results reported in previous studies have always been contradictory [28], [29]. Consequently, we performed the present meta-analysis to evaluate the relationships of common functional polymorphisms in the *ALDH2/ADH1/ADH2* genes with gastric carcinogenesis.

## Methods

### Search strategy

The PubMed, CISCOM, CINAHL, Web of Science, Google Scholar, EBSCO, Cochrane Library, and CBM databases were searched for relevant articles published before November 1st, 2013 without any language restrictions. The following keywords and MeSH terms were used: [“SNP” or “mutation” or “genetic polymorphism” or “variation” or “polymorphism” or “single nucleotide polymorphism” or “variant”] and [“gastric cancer” or “stomach cancer” or “gastric neoplasms” or “gastric cancer” or “gastric carcinogenesis” or “stomach neoplasms”] and [“acetaldehyde dehydrogenase 2” or “ALDH2” or “alcohol dehydrogenase II” or “alcohol dehydrogenase 1” or “alcohol dehydrogenase 2” or “ADH1” or “ADH2”]. We also performed a manual search of the reference lists from the relevant articles to find other potential articles.

### Selection criteria

The included studies must meet all four of the following criteria: (1) the study design must be clinical cohort or case-control study that focused on the relationships of *ALDH2/ADH1/ADH2* genetic polymorphisms with the pathogenesis of gastric cancer; (2) all patients diagnosed with gastric cancer must be confirmed through histopathologic examinations; (3) the genotype frequencies of healthy controls should follow the Hardy-Weinberg equilibrium (HWE); (4) the study must provide sufficient information about the genotype frequencies. If the study could not meet the inclusion criteria, it would be excluded. The most recent or the largest sample size publication was included when the authors published several studies using the same subjects. The supporting PRISMA checklist is available as supplementary information; see Checklist S1.

### Data extraction

Relevant data were systematically extracted from all included studies by two observers using a standardized form. The researchers collected the following data: language of publication, publication year of article, the first author's surname, geographical location, design of study, sample size, the source of the subjects, genotype frequencies, source of samples, genotyping method, evidence of HWE, etc.

### Quality assessment

Methodological quality was evaluated separately by two observers using the Newcastle-Ottawa Scale (NOS) criteria [30]. The NOS criteria included three aspects: (1) subject selection: 0∼4; (2) comparability of subject: 0∼2; (3) clinical outcome: 0∼3. NOS scores ranged from 0 to 9 with a score ≥7 indicating a good quality. The supporting NOS score criterion is available in Supplement S1.

### Statistical analysis

The STATA version 12.0 (Stata Corp, College Station, TX, USA) software was used for meta-analysis. We calculated crude odds ratios (ORs) with their 95% confidence intervals (95%CI) to evaluate their relationships under 5 genetic models [31]. Genotype frequencies of healthy controls were tested for the HWE using the *χ^2^* test. The statistical significance of pooled ORs was assessed by the *Z* test. The Cochran's *Q*-statistic and *I^2^* test were used to evaluate potential heterogeneity between studies [32]. If *Q*-test shows a *P*<0.05 or *I^2^* test exhibits >50% which indicates significant heterogeneity, the random-effect model was conducted, or else the fixed-effects model was used. We also performed subgroup analyses to investigate potential sources of heterogeneity. We conducted a sensitivity analysis to assess the influence of single studies on the overall ORs. Begger's funnel plots and Egger's linear regression test were used to investigate publication bias [33].

## Results

### Baseline characteristics of included studies

Initially, the searched keywords identified 132 articles. We reviewed the titles and abstracts of all articles and excluded 59 articles; full texts were also reviewed and 66 articles were further excluded. Finally, 7 case-control studies with a total of 2,563 gastric cancer patients and 4,192 healthy subjects met our inclusion criteria for qualitative data analysis [16], [24], [27]–[29], [34], [35]. Figure 1 shows the selection process of eligible articles. Distribution of the number of topic-related literature in electronic databases during the last decade is shown in Figure 2. Overall, six studies were conducted among Asians and only one study was performed among Caucasians. Nine common polymorphisms were evaluated, including rs671, rs16941667 and rs886205 in the *ALDH2* gene, rs1230025, rs13123099, rs698 and rs1693482 in the *ADH1* gene, and rs1229984 and rs17033 in the *ADH2* gene. Five genotyping methods were used in these studies, including PCR-RFLP, PCR-DHPLC, TaqMan assay, GoldenGate assay, and PCR-APLP methods. None of the studies deviated from the HWE (all *P*>0.05). NOS scores of all included studies were ≥5. We summarized the study characteristics and methodological quality in Table 1.

**Figure 1:** Flow chart of literature search and study selection. Seven case-control studies were included in this meta-analysis.

**Figure 2:** Distribution of the number of topic-related literatures in the electronic database during the last decade.

**Table 1:** Baseline characteristics and methodological quality of all included studies.

First author	Year	Country	Ethnicity	Sample size		Gender (M/F)		Age (years)		Genotyping method	Gene	SNP type	HWE test (*P* value)	NOS score
				Case	Control	Case	Control	Case	Control					
Matsuo et al [27]	2013	Japan	Asian	697	1372	521/176	1028/344	-	-	TaqMan array	*ALDH2*	rs671	0.294	7
Duell et al [16]	2012	France	Caucasian	364	1272	213/151	755/517	58.4±7.9	58.4±7.7	GoldenGate assay	*ADH1*	rs1230025	0.187	8
												rs13123099	0.869	
											*ALDH2*	rs16941667	0.080	
Shin et al [29]	2011	Korea	Asian	445	370	307/138	188/182	64.3±8.4	63.6±8.5	PCR-RFLP	*ALDH2*	rs886205	0.079	8
Ding et al [34]	2011	China	Asian	382	382	382/0	382/0	35∼85	-	PCR-DHPLC	*ADH2*	rs1229984	0.598	7
											*ALDH2*	rs671	0.240	
Zhou et al [35]	2010	China	Asian	201	199	201/0	199/0	65	65	PCR-DHPLC	*ADH2*	rs1229984	0.944	7
											*ALDH2*	rs886205	0.958	
Zhang et al [24]	2007	USA	Asian	305	428	-	-	-	-	TaqMan array	*ALDH2*	rs886205	0.172	6
											*ADH2*	rs1229984	0.633	
												rs17033	0.316	
											*ADH1*	rs698	0.068	
												rs1693482	0.522	
Yang et al [28]	2006	China	Asian	169	169	122/47	122/47	-	-	PCR-APLP	*ALDH2*	rs886205	0.759	6

Legend: M - male; F - female; SNP - single nucleotide polymorphism; HWE - Hardy-Weinberg equilibrium; NOS - Newcastle-Ottawa Scale; PCR-RFLP - polymerase chain reaction-restriction fragment length polymorphism; DHPLC - denaturing high performance liquid chromatography; APLP - amplified products length polymorphism.

### Quantitative data synthesis

Meta-analysis findings on the relationships of *ALDH2/ADH1/ADH2* genetic polymorphisms and gastric cancer risk were shown in Table 2. The results of our meta-analysis suggested that *ALDH2* genetic polymorphisms might be strongly correlated with an increased risk of gastric cancer (allele model: OR  = 1.21, 95%CI: 1.11∼1.32, *P*<0.001; dominant model: OR  = 1.23, 95%CI: 1.09∼1.39, *P* = 0.001; respectively) (Figure 3), especially for rs671 polymorphism. Furthermore, Furthermore, we observed significant associations between *ADH1* genetic polymorphisms and an increased risk of gastric cancer (allele model: OR  = 1.21, 95%CI: 1.08∼1.36, *P* = 0.001; dominant model: OR  = 10.52, 95%CI: 3.04∼36.41, *P*<0.001; respectively), especially for rs1230025 polymorphism. Among different ethnic subgroups, the results demonstrated positive correlations between *ALDH2/ADH1* genetic polymorphisms and an increased risk of gastric cancer among both Asians and Caucasians (Figure 4). Nevertheless, no positive relationships were found between *ADH2* genetic polymorphisms and gastric cancer risk (all *P*>0.05). The results of sensitivity analysis indicated that the overall pooled ORs could not be affected by single study (Figure 5). No evidence for asymmetry was observed in the Begger's funnel plots (Figure 6). Egger's test also failed to reveal any evidence of publication bias (all *P*>0.05).

**Figure 3:** Forest plots for the relationships of *ALDH2/ADH1/ADH2* genetic polymorphisms and the risk of gastric under the allele and dominant models.

**Figure 4:** Subgroup analyses of the relationships of *ALDH2/ADH1/ADH2* genetic polymorphisms and the risk of gastric under the allele model.

**Figure 5:** Sensitivity analysis of the summary odds ratio coefficients on the relationships of *ALDH2/ADH1/ADH2* genetic polymorphisms and the risk of gastric under the allele and dominant models.

**Figure 6:** Begger's funnel plot of publication biases on the relationships of *ALDH2/ADH1/ADH2* genetic polymorphisms and the risk of gastric under the allele and dominant models.

**Table 2:** Meta-analysis of the relationships of *ALDH2/ADH1/ADH2* genetic polymorphisms with the risk of gastric cancer.

	M allele vs. W (Allele model)			WM + MM vs. WW (Dominant model)			MM vs. WW + WM (Recessive model)			MM vs. WW (Homozygous model)			MM vs. WM (Heterozygous model)		
	OR	95%CI	*P*	OR	95%CI	*P*	OR	95%CI	*P*	OR	95%CI	*P*	OR	95%CI	*P*
***ALDH2*** ** gene**	1.21	1.11–1.32	<0.001	1.23	1.09–1.39	0.001	1.22	0.86–1.74	0.270	1.31	0.95–1.79	0.097	1.09	0.70–1.70	0.704
*SNP type*															
rs671	1.23	1.03–1.46	0.019	1.29	1.01–1.64	0.039	1.38	1.03–1.84	0.033	1.56	1.15–2.11	0.004	1.19	0.88–1.62	0.263
rs16941667	1.32	0.96–1.82	0.091	1.29	0.92–1.82	0.141	1.60	0.40–6.44	0.507	1.66	0.41–6.69	0.474	1.26	0.30–5.25	0.746
rs886205	1.13	0.98–1.30	0.085	1.15	0.96–1.38	0.137	1.05	0.51–2.15	0.895	1.09	0.61–1.95	0.775	0.97	0.39–2.42	0.941
*Ethnicity*															
Asians	1.20	1.08–1.33	<0.001	1.21	1.01–1.43	0.034	1.27	0.84–1.91	0.253	1.35	0.94–1.94	0.104	1.16	0.69–1.96	0.568
Caucasians	1.21	0.98–1.49	0.079	1.26	0.99–1.59	0.056	0.93	0.44–1.94	0.837	0.99	0.47–2.08	0.976	0.76	0.36–1.64	0.489
***ADH1*** ** gene**	1.21	1.08–1.36	0.001	10.52	3.04–36.41	<0.001	1.26	0.77–2.04	0.359	1.47	1.00–2.17	0.051	1.10	0.64–1.88	0.737
*SNP type*															
rs1230025	1.29	1.06–1.57	0.010	1.23	0.97–1.56	0.087	2.23	1.36–3.66	0.001	2.32	1.41–3.84	0.001	2.08	1.24–3.50	0.006
rs13123099	1.17	0.81–1.67	0.400	1.09	0.75–1.58	0.668	0.89	0.10–8.03	0.920	0.91	0.10–8.20	0.935	0.76	0.08–7.02	0.811
rs698	1.11	0.90–1.38	0.323	1.37	1.00–1.87	0.048	0.86	0.57–1.29	0.469	1.08	0.69–1.69	0.740	0.73	0.47–1.12	0.145
rs1693482	1.23	0.98–1.53	0.068	1.42	1.03–1.95	0.031	1.14	0.74–1.74	0.555	1.39	0.87–2.23	0.166	0.97	0.62–1.53	0.909
*Country*															
France	1.26	1.06–1.50	0.007	1.19	0.97–1.45	0.094	2.14	1.32–3.46	0.002	2.22	1.36–3.62	0.001	1.98	1.19–3.28	0.008
USA	1.17	1.00–1.36	0.048	1.39	1.12–1.74	0.003	0.98	0.73–1.32	0.905	1.22	0.88–1.68	0.232	0.84	0.61–1.14	0.256
***ADH2*** ** gene**	0.96	0.82–1.12	0.583	0.90	0.75–1.09	0.293	1.16	0.79–1.71	0.444	1.10	0.74–1.64	0.631	1.24	0.83–1.86	0.294
*SNP type*															
rs1229984	0.98	0.83–1.16	0.823	0.92	0.75–1.13	0.447	1.19	0.81–1.76	0.373	1.13	0.76–1.70	0.542	1.27	0.84–1.92	0.248
rs17033	0.79	0.50–1.25	0.320	0.80	0.50–1.30	0.374	0.47	0.05–4.50	0.509	0.46	0.05–4.41	0.498	0.55	0.05–5.56	0.614
*Ethnicity*															
Asians	0.99	0.83–1.19	0.945	0.93	0.74–1.17	0.555	1.18	0.75–1.85	0.484	1.11	0.67–1.83	0.689	1.27	0.84–1.92	0.261
Caucasians	0.84	0.61–1.16	0.302	0.84	0.60–1.18	0.317	0.72	0.12–4.15	0.711	0.70	0.12–4.08	0.695	0.84	0.14–4.98	0.845

Legend: W - wild allele; M - mutant allele; WW - wild homozygote; WM - heterozygote; MM - mutant homozygote; SNP - single nucleotide polymorphism; OR - odds ratio; 95%CI - 95% confidence interval.

## Discussion

The present meta-analysis indicated that *ALDH2* genetic variants were significantly correlated with the risk of gastric cancer, suggesting that these polymorphisms may be capable of modifying the susceptibility to gastric cancer. A biologically plausible explanation may be that genetic mutants in the *ALDH2* gene might diminish its enzyme activity which was suspected to be an important and strong protective factor against alcoholism by eliminating most of the toxic and carcinogenic acetaldehyde generated during alcohol metabolism [33]. The ALDH2, as a member of ALDH family, has been commonly regarded as a major mitochondrial metabolic enzyme that is strongly expressed in various tissues with the highest level of expression in the liver [36]. In recent years, epidemiological evidences have documented that genetic polymorphisms in *ALDH2* gene may play an important role in modifying the susceptibility to gastric cancer [37], [38]. ALDH2 exhibits a high activity for oxidation of acetaldehyde, which has been involved in the ethanol metabolic pathway, converting acetaldehyde to acetic acid, and plays a major role in acetaldehyde detoxification [39]. Genetic variants in *ALDH2* may cause an inability to metabolize acetaldehyde and conduce to the accumulation of acetaldehyde after alcohol intake, thereby inducing the occurrence of gastric cancer [20], [29].

We also observed that individuals with *ADH1* genetic polymorphisms were at a higher risk of developing gastric cancer, indicating that genetic variants in the *ADH1* gene might play a pivotal role in the pathogenesis of gastric cancer. The ADH1, belongs to the short chain ADH superfamily, is a glucose-repressible alcohol dehydrogenases which is crucial in the conversion of ethanol to its carcinogenic metabolite, acetaldehyde, particularly in the elimination phase, and is mainly expressed in the liver as well as gastric mucosa [40]. To date, there is evidence to suggest that the pathogenesis of gastric cancer may be greatly associated with acetaldehyde exposure [25]. Although the exact role of ethanol consumption in the development of gastric cancer is poorly understood and remains to be elucidated, it has been demonstrated that genetic variants in the *ADH1* gene may decrease its function or activity, and the less-active *ADH1* might lead to a decreased elimination rate of ethanol and result in prolonged exposure to microbially derived carcinogenic acetaldehyde, which may play an essential role in the pathogenesis of gastric cancer [12], [41].

However, we found no associations between *ADH2* genetic polymorphisms and gastric cancer risk, revealing that *ADH2* genetic polymorphisms may not be important dominants of susceptibility to gastric cancer. Although the role of *ADH2* genetic polymorphisms in the incidence of gastric cancer remains poorly understood yet, a probable reason for these results might be that *ADH2* genetic variants may enhance its activity which was responsible for formation of acetaldehyde by oxidating ethanol, while acetaldehyde has been postulated to be a factor that can intensify carcinogenesis [15]. Jelski et al. also reported that changes in the activity of ADH2 caused by genetic variants in gastric cancer patients seems to be induced by release of the isoenzyme from cancer cells [25].

The current meta-analysis also had many limitations that should be acknowledged. First, our results had lacked sufficient statistical power to assess the correlations between *ALDH2/ADH1/ADH2* genetic polymorphisms and the etiology of gastric cancer. Secondly, meta-analysis is a retrospective study that may lead to subject selection bias, and thereby affecting the reliability of our results. Thirdly, our meta-analysis failed to obtain original data from the included studies, which may limit further evaluation of potential role of *ALDH2/ADH1/ADH2* genetic polymorphisms in the development of gastric cancer. Although our study has several limitations, this is the first meta-analysis focusing on the correlations between *ALDH2/ADH1/ADH2* genetic polymorphisms and the pathogenesis of gastric cancer. Furthermore, we performed a highly sensitive literature search strategy for electronic databases. A manual search of the reference lists from the relevant articles was also conducted to find other potential articles. The selection process of eligible articles was based on strict inclusion and exclusion criteria. Importantly, rigorous statistical analysis of SNP data provided a basis for pooling of information from individual studies.

In conclusion, the current meta-analysis suggests that *ALDH2* and *ADH1* genetic polymorphisms may play crucial roles in the pathogenesis of gastric cancer. However, *ADH2* genetic polymorphisms may not be important dominants of susceptibility to gastric cancer. However, due to the limitations mentioned above, more researches with larger sample size are still required to provide a more reliable and representative statistical analysis precisely.

## Supporting Information

Checklist S1 **PRISMA Checklist.**
(DOC)

Supplement S1 **The Newcastle-Ottawa Scale for assessing methodological quality.**
(DOC)

Diagram S1 (DOC)
